The article "Research on the Method of Acquiring Customer Individual Demand Based on the Quantitative Kano Model" was published in 2022. Journal: Comput Intell Neurosci.

# Research on the Method of Acquiring Customer Individual Demand Based on the Quantitative Kano Model

**DOI:** 10.1155/2022/5052711

**Published:** 2022-04-11

**Authors:** Laihong Du, Hua Chen, Yadong Fang, Xiaowei Liang, Yujie Zhang, Yidan Qiao, Zhen Guo

**Affiliations:** ^1^School of Mechanical and Electrical Engineer, Xi'an Technological University, Xi'an 710021, China; ^2^School of Management, Xi'an University of Finance and Economics, Xi'an 710010, China

## Abstract

In order to realize accurate marketing by analyzing customer individual demand, a new quantitative Kano model method is put forward, and it is helpful to provide customized products for heterogeneous customer classification groups. By improving the traditional Kano model, the customer satisfaction and the importance degree of products are defined, and the quantitative Kano demand model is established. Customers are classified as the price preference group, the brand preference group, and the service priority group, and decision-making of product attribute quality improvement for customer classification is realized. Lastly, electric vehicles (EVs) are selected as a study case, and their various demands for different classifications of customers are discussed by questionnaire survey and calculation of satisfaction and the importance degree. Furthermore, different customer group demands are classified as attractive demands, expected demands, nondifferential demands, or essential demands, and the important product attribute acquisition process for various customers is discussed to improve enterprise market competitiveness.

## 1. Introduction

With the continuous improvement of people's consumption levels and the diversification of product forms, more and more consumers no longer simply pay for the premium of the product brand but expect to achieve consumption upgrading on the basis of the price, which also brings huge opportunities and challenges for enterprises to design and customization of products and services. Many manufacturing enterprises have also been user-centered, driven by the demand side, and depicted the user portrait on the basis of big data mining and analysis, so as to realize personalized customized services to users. As early as 1998, Yeh and Pearlson proposed the concept of customer customization, providing the corresponding personalized design, production, and delivery of customer products or services according to their personalized needs [1, 2]. Foreign IKEA and BMW-Mini have launched user customization in product customization, while Amazon, Haier, and other websites have made personalized recommendations for use [3]. Domestic red collar and WeiShang fully reflect the personalized personalization in the product application [4]. Enterprises can segment the market, regard the same type of users as a market segment, and provide them with the corresponding customized services to meet the personalized needs of users [5]. Personalized needs are to let products or services reflect their own unique needs and personality, not different needs from others. Therefore, while all users have common needs, the types of users can be distinguished through the personalized needs of users, and the products and services can be customized for different users' needs, which is of great significance to improving the competitiveness of enterprises in the same industry and the formation of precise marketing for customers.

At present, there is a certain vague uncertainty in the expression of user demand for products and services. How to maximize the personalized needs of users is the key to enterprise customization. There are two main ways to obtain information about users' needs: one is the data collection based on the Internet with the help of marketers. In [6], they proposed a method of product personalized customization with a case-based reasoning theory to solve the problem of low matching between user requirements and product modules in the process of product personalized customization. A new method for KANO model classification was created in [7]. By collecting customer reviews and rating scores, the author builds a regression model between the score and the degree to which product attributes meet user needs according to their text expression. However, the cost of one-to-one communication with customers is high, and the expression of product demands in the process of independent selection is vague. Besides, the existing options and parameters are difficult to meet the needs of customers. In [8], they researched the user's personalized needs of smart health preserving pot based on the Kano model to guide the interaction design and make the interaction of smart health preserving pot more fit the user's real needs. In [9], they focused on investigating traditional garment enterprises' transformation from mass production to mass customization, and it probed deeply into the ways for the garment manufacturing industry to realize Internet-based mass customization and key problems to be solved. An approach of integration of the Kano model into QFD to examine customer satisfaction based on aesthetic sentiments was proposed in [10], and a sport utility vehicle has been selected for the study. The aesthetic attributes have been selected with the help of QFD and their importance and classification have been calculated using both the fuzzy Kano and the traditional Kano models. [11]aimed to examine consumer perspectives about service satisfaction in the domestic medical industry using Kano's two-dimensional model and employed the importance-satisfaction model to determine service items that need improvement. In [12], they estimated customer preference based on conjoint analysis and categorized service quality elements by the IPA-Kano model. A methodology that integrates the Kano model (KM), analytic hierarchy process (AHP), and quality function deployment (QFD) methods with intuitionistic fuzzy set (IFS) to solve decision-making problems in new product development and design was proposed in [13]. By the new method, the web crawler technology was first applied to e-commerce web sites to collect raw data, and the representative CRs were extracted through combining the LDA model with the Apriori algorithm. Second, the intuitionistic fuzzy Kano model (IFKM) is proposed to evaluate the adjustment coefficient of CRs and Kano categories via customer preference membership functions. In [14], they proposed the product feature KANO analysis method based on the emotional distribution of product features, and Kano analysis of product characteristics by using product review data can provide valuable reference information for companies to improve their products. Literature [15] classified the product functions mentioned in social media. In [16], they divided the design demands information of personal protective mask into several attributes initially and obtained the final Kano required attributes by the better-worse coefficient analysis method. In [17], they used the Kano model to identify and screen demand and built the quality demand hierarchy model of high-quality housing to calculate the importance degree of each demand item. In the study [18], they defined the user requirements in the Kano model and classified user requirement hierarchies using the rough analysis hierarchy process method to calculate requirement weight. In [19], a hybrid Kano model with tools of SII and DDI was proposed.

Most of the existing customer demand determination methods are to calculate the importance degree of a customer's personalized demands and then determine the priority of the customer's demands, ignoring the existence of product satisfaction. Product satisfaction is an important and influencing factor of product upgrading, and it can realize product accuracy in marketing if the demands of customers are quantified with feedback on product importance and satisfaction. Therefore, this paper acquires the customer preferences for different types of demands by through a quantified Kano model classification according to the importance degree of customer demands. Furthermore, the satisfaction and importance evaluation of customer demands are combined to determine which types of demand items should be emphasized in the later update and upgrading of products so as to provide user groups with products that meet customer scenarios and actual demands in the future.

## 2. Related Work

The Kano model was formally proposed by Japanese scholar Yoshino. According to the subjective performance of the product and the customer subjective perception [11], the quality characteristics of the product were classified and screened. Among them, the customer's demand for products is divided into five categories, namely, necessity, expectation, charm, no difference, and reverse [20]. Must-be requirement refers to the basic requirements that the product should have. If the attribute is sufficient, the user will not be delighted, but if the point is absent, the user will be very dissatisfied. Attractive requirement, also known as excited demand, is a characteristic that can surprise or surprise customers. When it is sufficient, it can improve customer satisfaction to a large extent, but it will not cause dissatisfaction when it is insufficient. One-dimensional requirement is an essential factor for enterprises to evaluate competitiveness, which makes customers satisfied when the product has enough characteristics and causes dissatisfaction when it is not sufficient. Indifferent requirement, customers ignore factors, and whether it is satisfied does affect users' satisfaction with products. Reverse requirement, when product attributes are satisfied, customers are not satisfied, and when product attributes are not satisfied, customers are more satisfied. According to the objective performance of the product and customer satisfaction, the Kano model diagram is shown in Figure 1.

The Kano model requirement classification evaluation table designs the product attributes as positive and negative aspects and obtains the demand classification of product attributes by analyzing the Kano questionnaire filled by users. Among them, *M* represents the necessary demand, O represents the expected demand, A represents the charming demand, I represents the nondifference demand, *R* represents the reverse demand, and *Q* represents the problem demand (Table 1).

The traditional Kano model is essentially a qualitative analysis method, and its classification method is subjective. The preference of product characteristics is classified by the degree of selection of positive and negative problems in the Kano model demand classification evaluation table, which lacks quantitative standards. Therefore, it is of great significance to quantitatively improve the traditional Kano model and divide the user's demand preference after quantification, so as to realize the precise marketing of users.

## 3. Quantitative Kano Model Method

Different people have different demand expectations for the same product. The type of demand item can be determined according to the user's satisfaction degree and the importance degree of product services. Unlike the traditional Kano demand acquisition model, the quantitative Kano model will measure the user's expectation of the product through quantitative indicators, which can more objectively obtain the user's personalized demands.

The initial personalized hierarchical model is constructed. The quantitative Kano model is used to divide the initial demand according to the satisfaction index to determine the personalized demand category. Due to the heterogeneity of users, users are divided into different types. Users' evaluation of the importance of product services is added to improve the quality of personalized demands further and finally obtain the personalized priority demands of heterogeneous users. Getting personalized orders of heterogeneous users can be summarized in Figure 2.

The basic idea of quantifying users' satisfaction degrees and the importance degree of product service is as follows:

**Step 1 .**

Identify the initial personalized demand level.

The product specification is checked, and the relevant literature is read to understand the product characteristics that may be customized. At the same time, through face-to-face interviews with the sales staff, technicians, and customers, the requirements are obtained that the customer in the purchase process may mention the product. The original requirements are analyzed, deleted, and modified. The concept scope of the product is broad in the product instructions and interviews. The concept can be hierarchically sorted and summarized according to the affinity graph method, and Figure 3 of the initial personalized demand hierarchy model of the product is constructed (*PR* = {*PR*_*1*_, *PR*_*2*_, *PR*_*i*_,...,*PR*_*n*_}, *PR*_*i*_ _*=*_ {*PR*_*i1*_, *PR*_*i2*_, *PR*_*ik*_,...,*PR*_*is*_}).

**Step 2 .**

Design of a quantitative Kano questionnaire.

Combined with Matzler's research, numerical indicators are set up in the user's product service satisfaction degree and importance degree. The user's demand options are quantified and counted when analyzing the questionnaire. At the same time, the quantitative Kano model is applied to different user groups, and the Kano demand types corresponding to different kinds of user groups are analyzed.

Because the positive answer is stronger than the negative answer, the index scale of satisfaction degree asymmetry can be set in the questionnaire to reduce the influence of negative evaluation and obtain the corresponding quantitative values for different personalized demands [12]. In addition, the importance degree of product services is divided into four degrees, the value is divided according to different levels, and the corresponding quantitative range is formulated. The Kano model requirements for classification evaluation table quantification criteria are shown in Tables 2 and 3.

**Step 3 .**

Calculation of customer satisfaction with product services.

**Step 31 .**

Assume variables.

According to the quantitative Kano model designed by the questionnaire data analysis,

Assume *V* represents a set of users, and *v*_*j*_ represents the *j*th user.

(1) $$\begin{array}{c} V=\left\{v_{j}|j=1,2,\ldots ,n\right\}. \end{array}$$

Assume *F* represents a collection with product service attributes, and *f*_*i*_ represents the *i*th product service attribute.

(2) $$\begin{array}{c} F=\left\{f_{i}|i=1,2,\ldots ,m\right\}. \end{array}$$

Assume that *x*_*ij*_ is the reverse product service satisfaction evaluation of *j*th users when the product service attribute *f*_*i*_ is not provided. *y*_*ij*_ is the positive product service satisfaction evaluation of user *j* when providing product service *f*_*i*_. *ω*_*ij*_ is the importance evaluation of user *j* on product service attribute *f*_*i*_. For each user *v*_*j*_, the evaluation of *f*_*i*_ can be expressed as follows:

(3) $$\begin{array}{c} e_{ij}=\left(x_{ij},y_{ij},\omega_{ij}\right). \end{array}$$

**Step 32 .**

Calculate the average value of users' positive and negative problems.

By designing a quantitative Kano questionnaire, the values of *x*_*ij*_, *y*_*ij*_, and *ω*_*ij*_ can be obtained by questionnaire analysis. ${\bar{X}}_{i}$ denotes the average level of user satisfaction with negative problems without providing *f*_*i*_ product service attributes; ${\bar{Y}}_{ij}$ represents the average level of user satisfaction with a forward problem when providing *f*_*i*_ product service attributes, which are as follows:

(4) $$\begin{array}{c} {\bar{X}}_{i}=\frac{1}{n}\sum_{j=1}^{n}\omega_{ij}x_{ij},\\ {\bar{Y}}_{i}=\frac{1}{m}\sum_{i=1}^{m}\omega_{ij}y_{ij}. \end{array}$$

The value of $\left({\bar{X}}_{i},{\bar{Y}}_{i}\right)$ can be marked in the two-dimensional coordinate diagram. The abscissa is the user's dissatisfaction with the product service attribute *f*_*i*_, and the ordinate indicates the satisfaction level. Most $\left({\bar{X}}_{i},{\bar{Y}}_{i}\right)$ values fall within the range of [0, 1] in the two-dimensional graph, and the negative value is reverse demand or problem demand, which is not included in the average value, as shown in Figure 4.

**Step 33 .**

Calculate the user product service importance degree and satisfaction degree index.

Product service attributes can be described as $f_{i}∼{\overset{⟶}{r}}_{i}=\left(r_{i},a_{i}\right)$ in vector form, where *r*_*i*_ is the moment of vector $\vec{r_{i}}$, which represents the importance of the product service attribute *f*_*i*_ to the user and is the Kano importance degree index.

(5) $$\begin{array}{c} r_{i}=\left|{\overset{⟶}{r}}_{i}\right|=\sqrt{{\bar{x}}_{i}^{2}+{\bar{y}}_{i}^{2}},\;0\leq r\leq \sqrt{2}, \end{array}$$

where *a*_*i*_ is the angle between the vector $\vec{r_{i}}$ and the horizontal coordinate axis, which determines the relative level of user satisfaction or dissatisfaction with the product service attributes and becomes the Kano satisfaction index.

(6) $$\begin{array}{c} \alpha_{i}=\text{arctg}\left(\frac{\bar{Y}i}{{\bar{X}}_{i}}\right),\;0\leq \alpha_{i}\leq \frac{\pi }{2}. \end{array}$$

**Step 4 .**

Decision on quality improvement of product service.

According to the quantitative Kano questionnaire, the user demands are divided into attractive demands, essential demands, expected demands, and nondifference demands, and the user groups filled in the questionnaire are classified. At the same time, the importance of product services filled out by users in the questionnaire is used to further improve the quality of personalized demand for product services. Taking Kano satisfaction degree and Kano importance degree as two dimensions, product service attributes are divided into four quadrants. As shown in Figure 5, $\bar{r}$ is the average value of product service attributes importance degree, and $\bar{\partial }$ is the average value of product service satisfaction degree.

According to the analysis of Figure 5, quadrant I can be summarized as an irrelevant region. The product service attributes of the region have little effect on customer satisfaction and importance degree. Enterprises do not need to spend too many resources to improve these attributes. Quadrant II is the oversatisfaction area. Customers have high satisfaction with the product service in the region, but the importance of this attribute is not high. Investment in the region's attributes can be moderated if companies demand to reduce costs. Quadrant III can be regarded as a performance improvement area, which has high satisfaction and an important degree of product and service attributes. Increasing investment in this regional details can improve customer satisfaction. Quadrant IV can be classified as a key promotion area, and it has a low satisfaction degree and a high importance degree. It shows that the product service attributes in the region play a significant role in user demands. If customer satisfaction with these attributes can be improved, the quality requirements of product services can be improved as a whole.

## 4. Case Study

Taking electric vehicles as an example, this paper establishes the initial demand item model of the electric vehicle, subdivides the customizable part of the electric vehicle, and determines the demand item problem of the quantitative Kano questionnaire. The personalized customization needs of different types of user groups for electric vehicles are obtained through a questionnaire. The quantitative Kano analysis method is used to quantify the satisfaction and importance of users to products and services. Then, the demand items are divided into corresponding types so that enterprises can carry out precision marketing for different demand types of heterogeneous users.

### 4.1. Construction of Initial Requirements Model for Electric Vehicle

The collected electric vehicle demand items are divided into four categories: internal appearance demand, software and hardware demand, functional demand, and service demand. Among them, the internal and external demand refers to the internal and external decoration, including the vehicle's external characteristics and internal design. The design of this part reflects the user's demand for the overall beauty and comfort of the vehicle. The software and hardware requirements involve the vehicle's software and hardware systems, which can ensure the safety of vehicle performance and the intellectualization of the system. Functional requirements include entertainment, transmission, and additional functions. These functions can satisfy users and meet users' expectations for the vehicle. The service demand can be used as the value-added service of the product. While providing users with product functions, the existence of these functions will make users more satisfied and enhance the value of the product. Therefore, the construction of the initial demand model of electric vehicles is shown in Figure 6.

### 4.2. Design of the Quantitative Kano Questionnaire

The questionnaire is designed based on the initial personalized demand hierarchy model of electric vehicles. The questionnaire is divided into two parts. The first part is to investigate the characteristics of customers and establish the relevant preferences of customers. The second part is designed in the form of selection (positive and negative problems) and filling (importance degree). The customers' EV demand items are shown in Table 4.

### 4.3. Analysis of Electric Vehicle Demand Items of Users

Combined with the Kano demand questionnaire of EV and Equations 1–4, the negative and positive satisfaction degree distribution is shown in Figure 7 and Figure 8. There are three customer groups and 25 demand items, and the satisfaction degrees of various preference customers and demand items are different. The results in Figures 7 and 8 demonstrate that the negative satisfaction degree of demand item *f*_14_ (wheel hub) is the highest, and the positive satisfaction degree of demand item *f*_11_ (connection of vehicle networking data) is the highest.

In terms of the statistical results in the previous table, the satisfaction threshold is set to 0.5 for the product service attribute *x*_*i*_ < 0.5, *y*_*i*_ < 0.5 is divided into no difference. If *x*_*i*_ ≥ 0.5, *y*_*i*_ < 0.5 is classified as an essential requirement. When *x*_*i*_ ≥ 0.5, *y*_*i*_ ≥ 0.5, it is considered an expected demand. Similarly, when *x*_*i*_ ≤ 0.5, *y*_*i*_ ≥ 0.5 can be divided into charismatic needs. Based on the abovementioned settings, by depicting the data in Figures 7 and 8, we can get the average satisfaction to scatter diagram of all users and different user groups on product service attributes. Different user groups are price advantage users, brand affects users, and service users before and after sales.

According to the scatter diagram in Figure 9, for the samples of all users, the size of trunk space, the setting of the speech recognition system, and the additional products of the vehicle are divided into charm requirements. The four attributes of battery life function, data connection of the Internet of vehicles, exclusive manual customer service, and remote charging are divided into expected requirements. Eight choices, including the choice of seat configuration, car suspension choice, and GPS positioning and navigation system, can be divided into necessary requirements. The other ten attributes, such as the customization of the vehicle color, the selection of sunroof type, and the type of key, can be classified as indifference requirements.

According to the heterogeneity characteristics of users, the perception of the same product service attributes is also different. Users can be subdivided into heterogeneous user groups. According to the description of the scatter diagram, the demand types of users can be classified and summarized according to different groups, and the following product service attributes (Table 5) of heterogeneous user groups about electric vehicles can be obtained.

It can be found from Table 5 that different user groups have heterogeneity on product and service attributes, and user stickiness and market influence can be enhanced by providing users with differentiated, personalized product and service attributes. For user groups that prefer price advantage, their user groups pay more attention to the cost performance of products and expect to use the least money to obtain higher quality products and services. They do not have too much expectation for products and services and can meet their basic needs. For the user groups that prefer brand effect, their users pay more attention to the product and service guarantees brought by the product brand and think that the greater the brand influence, the better the effectiveness of their products and services. Such subdivided users have higher standards for the attributes of products and services and expect the attributes of the products and services they use to pass the high-quality screening. This is consistent with the characteristics of the user preference brand effect. User groups who prefer sales services pay attention to the services provided in purchasing products and the sense of the experience of process services. The humanized services of user enterprises often move such users.

To sum up, users have heterogeneous characteristics for user groups with different purchase preferences. Considering the different needs of heterogeneous users, the classification of the same product and service attributes will also belong to different demand types. Enterprises can pay attention to the expected needs of heterogeneous user groups. Everyday needs are the key for enterprises to improve their competitiveness. Providing personalized, customized services for different users can effectively improve user satisfaction and stickiness to enterprise products and services.

### 4.4. User Demand Promotion Decision

According to the personalized needs of heterogeneous users, the quality of their product service attributes can be improved accordingly. The $\left|{\overset{⟶}{r}}_{i}\right|$ and *α*_*i*_ values of all users and heterogeneous user groups are calculated. Electric vehicles product and service attributes are classified into four quadrants composed of demand, satisfaction, and importance. The distribution of various demands of overall customers is shown in Figure 10, and the quantitative Kano model decision matrix of customers who prefer price is illustrated in Figures 11.  Figure 12 describes the demand distribution of customers who prefer brand, and the quantitative Kano model decision matrix of customers who prefer service is shown in Figure 13.

According to the importance of demand attributes, the third quadrant and the fourth quadrant can be divided into performance improvement areas and critical improvement areas. The abovementioned figure shows that whether all users or different types of users, the demand attributes of the third and fourth quadrants are mostly necessary needs and expected needs. On the one hand, it expresses that good products can not only meet the most basic needs of users but also pay attention to the expected needs, that is, pay attention to the core competitiveness of enterprises, which is consistent with the classification of the quantitative Kano model mentioned above, which verifies the necessity of user demand classification. The product service attributes can be improved according to the quality decision matrix obtained from the product service satisfaction and importance, and precise marketing can be carried out according to the user's pain points.

## 5. Conclusion

In the traditional Kano model, customer demand items are determined according to statistics of positive and negative problems that customers had with product attributes, and it ignores various customer demand classifications. Furthermore, the traditional Kano model leads to subjective demand classification results for its qualitative selection. Satisfaction and importance degree of customers are put forward to judge different demand preferences of different customers for the same product by the quantitative Kano model, and it is helpful to realize precise marketing of the product. The paper takes electric vehicles as an example. An initial demand model of product is first constructed, and then customer demand items are determined. It can get a quantitative perception evaluation of electric vehicle satisfaction and importance degree by the Kano demand questionnaire and Equations 1–5, and the result shows that it can improve demand matching quality. For heterogeneous customers, each product attribute may belong to various demand types. In the process of customer purchase, enterprises should focus on customer's expected demands and essential demands, which will change with different types of customers. The quality of those demands will affect the customer's purchase choice. At the same time, the research results can be applied to the process of customer demand type determination and demand quality decision-making in various industries, which is helpful to the enterprise demand management and upgrading for the corresponding customer. The focus of the further research in the paper is to transmit customer demands into EV product functions based on ontology technology.

## Figures and Tables

**Figure 1:** Kano model schematic.

**Figure 2:** Process of obtaining personalized requirements for heterogeneous users.

**Figure 3:** Initial hierarchy model of personalized requirements.

**Figure 4:** Quantitative standards for product and service requirements.

**Figure 5:** Decision on quality improvement of product service attributes.

**Figure 6:** Construction of initial demand model of electric vehicle.

**Figure 7:** Negative satisfaction degree *x¯*_*i*_ statistical analysis of electric vehicle individual demand.

**Figure 8:** Positive satisfaction degree *y¯*_*i*_ statistical analysis of electric vehicle individual demand.

**Figure 9:** Scatter chart of mean satisfaction of overall customers with product attributes.

**Figure 10:** Quantitative Kano model decision matrix of overall customers.

**Figure 11:** Quantitative Kano model decision matrix of customer who prefer price.

**Figure 12:** Quantitative Kano model decision matrix of customers who prefer brand.

**Figure 13:** Quantitative Kano model decision matrix of customers who prefer service.

**Table 1:** Kano model demand classification evaluation table.

Positive problem	Reverse problem				
	Like	Naturally	Never mind	Passable	Dislike
Like	Q	A	A	A	O
Naturally	R	I	I	I	M
Never mind	R	I	I	I	M
Passable	R	I	I	I	M
Dislike	R	R	R	R	Q

**Table 2:** Provision/nonprovision of satisfaction values for product and service attributes.

		Like	Naturally	Never mind	Passable	Dislike
Product attributes	Provides this attribute	1	0.5	0	−0.25	−0.5
	This attribute is not provided	−0.5	−0.25	0	0.5	1

**Table 3:** Importance degree of products and services.

Unimportant	Some important	Important	Very important
0–0.25	0.25–0.5	0.5–0.75	0.75–1

**Table 4:** Description of product/service attributes of electric vehicles.

Product/service attribute number	Product/service attribute number	Benefits for users
*f*_*1*_	Custom vehicle colors	Personality and pleasure
*f*_*2*_	The type of sunroof can be selected	Comfortable and safe
*f*_*3*_	Selection of seat configuration	Comfortable and safe
*f*_*4*_	Size adjustment of trunk space	Convenient and comfortable
*f*_*5*_	Battery life function	Value-added and convenient
*f*_*6*_	Type of key	Personality and convenience
*f*_*7*_	Selection of onboard purification equipment	Safe and comfortable
*f*_*8*_	Choice of automobile suspension	Personality and safety
*f*_*9*_	Customization of entertainment functions	Personality and pleasure
*f*_*10*_	The setting of the speech recognition system	Fast and convenient
*f*_*11*_	Connection of vehicle networking data	Safe and fast
*f*_*12*_	Selection of GPS positioning and navigation system	Personality and convenience
*f*_*13*_	Vehicle additional products	Personality and value-added
*f*_*14*_	Wheel hub	Personality and safety
*f*_*15*_	Exclusive manual customer service	Added value and pleasure
*f*_*16*_	Maintenance service	Fast and safe
*f*_*17*_	Remote charging	Fast and value-added
*f*_*18*_	Copilot emergency system	Safe and convenient
*f*_*19*_	Intelligent parking	Fast and convenient
*f*_*20*_	Automatic driving	Fast and convenient
*f*_*21*_	Rear seat TV	Comfortable and pleasant
*f*_*22*_	Hi-Fi equipment	Comfortable and pleasant
*f*_*23*_	Lamp type	Personality and safety
*f*_*24*_	Vehicle shape	Personality and value-added
*f*_*25*_	Car refrigerator	Comfortable and pleasant

**Table 5:** Classification and summary of product/service requirements of heterogeneous users.

Product/service attributes	Users who prefer price advantage (73)	Users who prefer brand effect (66)	Users who prefer sales services (53)	All users (192)
*f*_*1*_	I	A	I	I
*f*_*2*_	I	I	I	I
*f*_*3*_	M	M	M	M
*f*_*4*_	A	A	A	A
*f*_*5*_	O	O	O	O
*f*_*6*_	I	I	I	I
*f*_*7*_	I	I	I	I
*f*_*8*_	M	M	M	M
*f*_*9*_	M	M	M	M
*f*_*10*_	A	A	A	A
*f*_*11*_	O	O	A	O
*f*_*12*_	M	O	M	M
*f*_*13*_	A	O	A	A
*f*_*14*_	M	M	M	M
*f*_*15*_	O	O	O	O
*f*_*16*_	M	M	O	M
*f*_*17*_	O	A	O	O
*f*_*18*_	I	I	I	I
*f*_*19*_	I	I	O	I
*f*_*20*_	I	I	I	I
*f*_*21*_	I	I	R	I
*f*_*22*_	M	O	M	M
*f*_*23*_	M	M	M	M
*f*_*24*_	I	A	I	I
*f*_*25*_	I	I	I	I

## Data Availability

The labeled dataset used to support the findings of this study are available from the corresponding author upon request.
